The article "OX40-Fc Fusion Protein Alleviates PD-1-Fc-Aggravated Rheumatoid Arthritis by Inhibiting Inflammatory Response" was retracted in 2023. Reasons: signs of a paper mill; suspected computer-generated content; unreliable results or conclusions; concerns about the data.

# OX40-Fc Fusion Protein Alleviates PD-1-Fc-Aggravated Rheumatoid Arthritis by Inhibiting Inflammatory Response

**DOI:** 10.1155/2022/6244175

**Published:** 2022-02-17

**Authors:** Yanyan Huang, Shudian Lin, Feng Zhan, Lu Xiao, Yuwei Zhan, Ru Wang

**Affiliations:** Department of Rheumatism and Immunity, Hainan General Hospital (Hainan Affiliated Hospital of Hainan Medical University), Haikou, Hainan 570311, China

## Abstract

**Background:**

Researches have confirmed that the abnormal signals of OX40 and PD-1 lead to the changes of T cell biological behavior, thus participating the immunopathological process of RA. However, the pathogenesis of RA immunopathological process has not been clarified yet.

**Methods:**

30 DBA/1 mice were randomly divided into 5 groups (6 mice per group): control group, collagen-induced arthritis (CIA) group, PD-1-Fc/CIA group, OX40-Fc/CIA group, and PD-1-Fc + OX40-Fc/CIA group. The pathological changes in mice joints were observed by H&E staining. The proportion of CD4+ T, CD8+ T, CD28+, and CD19+ cells in peripheral blood mononuclear cells (PBMCs) was detected by flow cytometry. Serum inflammatory factors (CRP, IL-2, IL-4, IL-1*β*, INF-*γ*) and bone metabolism-related genes (CTX-I, TRACP-5b, BALP) were detected by ELISA assay. Western blotting was applied to measure the NF-*κ*B signaling pathway-related protein (p-IKK*β*, p-I*κ*B*α*, p50) expression in synovial tissue of mice joint.

**Results:**

Compared with the control group, CIA mice showed significant increases in arthritis score and pathological score. In the CIA group, a marked decrease was identified in the proportion of CD8+ T, CD19+, and CD68+ cells. Additionally, the CIA group was associated with upregulation of secretion of inflammatory factors in serum and expression of bone metabolism-related genes and NF-*κ*B pathway-related proteins. Compared with the CIA group, the same indexes above showed a further aggravation in the PD-1-Fc group while all indexes improved in the OX40-Fc group. Besides, OX40-Fc fusion protein slowed down significantly the further deterioration of CIA mouse pathological process caused by PD-1-Fc fusion protein.

**Conclusion:**

OX40-Fc fusion protein alleviates PD-1-Fc-aggravated RA by inhibiting inflammatory response. This research provides biological markers with clinical significance for diagnosis and prognosis of RA, as well as offers theoretical and experimental foundation to the new targets for immune intervention.

## 1. Introduction

Rheumatoid Arthritis (RA) is a systemic autoimmune disease, with chronic progressive joint lesions as its main symptom [1]. The prevalence of RA is 0.32%-0.36% in China, which is slightly lower than the world average, and the incidence rate of male and female is about 1 : 3 [2, 3]. The main clinical manifestations of RA are symmetric polyarthritis, pain and swelling of hands, wrists, elbows, knees and foot joints, and morning stiffness [4]. Extra-articular manifestations of patients are fever, anemia, subcutaneous nodules, vasculitis, pericarditis, lymphadenopathy, and so on. And a variety of autoantibodies such as rheumatoid factor (RF), anti-cyclic citrullinated peptide antibody (anti-CCP antibody), and anti-keratin antibody (AKA) could be found in the serum in RA patients [5]. Without proper treatment, RA, along with persistent pain, can cause joint deformity and functional loss eventually. It seriously endangers patients' physical and mental health and affects their quality of life a lot. RA is a kind of autoimmune connective tissues disease characterized by massive infiltration of lymphocyte in chronic synovitis [6].

The article "OX40-Fc Fusion Protein Alleviates PD-1-Fc-Aggravated Rheumatoid Arthritis by Inhibiting Inflammatory Response" was retracted in 2023. Reasons: signs of a paper mill; suspected computer-generated content; unreliable results or conclusions; concerns about the data.

The pathogenesis of RA is complicated, which involves genetic, environmental, and immune factors [7]. And the immunopathological mechanism of RA mainly displays as T cell-mediated autoimmune disease. In the autoimmune process of RA, inflammatory T cells, B cells, macrophages, and dendritic cells infiltrate the joint synovium; then, interaction between cells leads to the occurrence of autoantibodies and the secretion of proinflammatory cytokines [8]. The expression of colony stimulating factors, chemokines, and adhesion molecules recruited macrophage-like synovial cells and osteoclasts, and then the joint structure was destroyed [9, 10]. And CD4+ helper T cells (hereafter called Th) play an important role in the immunopathology of RA, including Th1, Th2, and Th17 cells [11–13]. Recent studies have also found that there are abnormally elevated CD4+ CD28-T cell subsets in RA, which are continuously activated in a non-CD28 dependent manner. These CD4+ CD28-T cell subsets are characterized by long-term survival and clonal expansion, which are regarded as self-reactive effector memory T cells [14].

In the process of immune response, T cell activation not only needs the main histocompatibility complex- (MHC-) antigen peptide but also needs the collaborative participation of some other costimulation molecules, and among them, OX40/OX40L is a new costimulation molecule that has attracted much attention in recent years [15]. OX40 is a type I transmembrane glycoprotein in the TNFR family [16]. And OX40-mediated costimulation signals have a major part in the primary and secondary immune responses of T cells. These signals can promote the activation, proliferation, and migration of CD4+ T cells and prolong their life, as well as can accelerate the formation of germinal centers and the differentiation and maturation of cells [15, 17]. The OX40 expression is associated with specific T cells activated by antigen. Its biological function is to strengthen and maintain the specific immune response of effector specific T cells to antigen-specific effector [18]. The particularity of the OX40 expression and biological function makes it an ideal immune intervention target [19]. Different intervention measures are adopted for the mutual interaction between OX40 and its ligand. These intervention measures may be one of the effective methods to improve or inhibit immune response and treat RA diseases [20, 21]. Related studies have indicated that the loss or blocking of PD-1 signal can lead to autoimmune diseases [22]. Guo et al. has found that RA patients expressed PD-1 on a majority of synovial tissues infiltrating CD4+ and CD8+ T cells [23]. These studies suggest that the abnormal signals of OX40 and PD-1 are involved in the immunopathological process of RA. Huang et al. [24] have confirmed that the PD-1 and OX40 expression was observably elevated in CD4+ T lymphocytes that were separated from the peripheral blood and synovial fluid of RA patients and the spleen of collagen-induced arthritis (CIA) mice. Besides, OX40 can reverse all RA process caused by PD-1-Fc, but the mechanism is not clear. Therefore, this paper intends to utilize OX40-Fc fusion protein (OX40-Fc) to intervene CIA mouse and then evaluate the effects of this fusion protein on RA-induced immune imbalance and inflammatory factor secretion after a series of experiments; finally, according to the result, possible mechanism of anti-RA is explored.

The article "OX40-Fc Fusion Protein Alleviates PD-1-Fc-Aggravated Rheumatoid Arthritis by Inhibiting Inflammatory Response" was retracted in 2023. Reasons: signs of a paper mill; suspected computer-generated content; unreliable results or conclusions; concerns about the data.

## 2. Materials and Methods

### 2.1. Establishment and Grouping of the CIA Mouse Model

30 male DBA/1 mice (8-10 weeks) were conducted adaptive feeding for 2-3 days. Then, they were allocated randomly to the following 5 groups (6 mice/group): (1) no any treatment in the control group; (2) mice in the CIA group [25] were injected subcutaneously 100 *μ*L bovine type II collagen and 100 *μ*L complete emulsion of Freund's complete adjuvant at dorsal root for primary immune response. After 21 days, the same method was used to strengthen immunization. After strengthening immunity, normal saline was injected intraperitoneally once every 3 days; (3) CIA mice were intraperitoneally injected with PD-1-Fc once every 3 days after enhancing immunization in the PD-1-Fc group; (4) CIA mice were intraperitoneally injected with OX40-Fc once every 3 days after strengthening immunization in the OX40-Fc group; (5) CIA mice were intraperitoneally injected with PD-1-Fc and OX40-Fc once every 3 days after strengthening immunization in the PD-1-Fc + OX40-Fc group. This study was approved by the Animal Ethics Committee of Hainan General Hospital ([2020]-158).

The article "OX40-Fc Fusion Protein Alleviates PD-1-Fc-Aggravated Rheumatoid Arthritis by Inhibiting Inflammatory Response" was retracted in 2023. Reasons: signs of a paper mill; suspected computer-generated content; unreliable results or conclusions; concerns about the data.

### 2.2. Observation of Joint Score

From primary immune response, the activities, consciousness and redness, and swelling of paws of mice were observed. Swollen ankles were measured using digital calipers. The swelling of each paw was scored from 0 to 4 as follows [26]: 0, no swelling; 1, slightly swelling in toe joint and inflammatory reaction in a single area of toes or pads; 3, swelling extending to metatarsal joints and toes below the ankle, moderately red swelling in joints, and mild dysfunction was caused; and 4, swelling extending to all pads and toes, including the ankle, with severe redness, swelling, stiffness, and even deformity of joints, and serious dysfunction was caused. The scores from each claw were added to get a total score between 0 and 16.

### 2.3. H&E Staining

Firstly, the ankle joint was fixed with neutral formic acid solution, and then decalcification was conducted. Subsequently, after longitudinal incision, the ankle joint was embedded in paraffin, then sectioned, and stained. After that, inflammation of the joint was observed: (1) pathological blind method was utilized to evaluate inflammatory cell infiltration: (1) centriole, lymphocyte, and plasma cell infiltration; (2) synovial cell proliferation, and fibrous tissues proliferation; and (3) cartilage and bone erosion; (2) synovitis was evaluated with following scores: 0 = no synovial inflammation, 1 point = local inflammatory infiltration, and 2 points = significant lymphocyte infiltration and synovial edema; and (3) the score of blood vessel and articular cartilage destruction was evaluated with following criteria: 0 = normal; 1 point = synovial hyperplasia attached to cartilage, but did not cause any damage to cartilage; and 2 points = synovial hyperplasia caused damage to cartilage.

### 2.4. Flow Cytometry

According to the instructions of the separation solution of peripheral whole blood mononuclear cells (PBMC, Solarbio, China), gradient centrifugation was used to obtain PBMCs in each group. Subsequently, 2 × 10^6^ separated PBMCs were stained, and then fluorescent dye labeled CD4, CD8, CD28, and CD19 monoclonal antibodies (BD Bioscience, USA) were added, respectively, after that they were incubated with light avoidance at 4°C for 30 min. Besides, corresponding isotype control antibodies were set with light avoidance incubation for 45 min. Subsequently, all antibodies were washed for 3 times by PBS. After that, flow cytometry was applied to analyze the result.

### 2.5. Enzyme Linked Immunosorbent Assay (ELISA)

According to the instructions of CRP, IL-2, IL-4, IL-1*β*, and INF-*γ* detection kits (R&D Systems), mouse serum samples were collected. By enzyme-linked immunosorbent assay, absorbance value was read at 540 nm wavelength. Then, the concentration of CRP, IL-2, IL-4, IL-1*β*, and INF-*γ* was calculated according to the standard curve.

The article "OX40-Fc Fusion Protein Alleviates PD-1-Fc-Aggravated Rheumatoid Arthritis by Inhibiting Inflammatory Response" was retracted in 2023. Reasons: signs of a paper mill; suspected computer-generated content; unreliable results or conclusions; concerns about the data.

The synovial tissues of mice were collected, and after homogenate, the cell suspension was collected. The levels of CTX-I, TRACP-5b, and BALP were measured by CTX-I, TRACP-5b, and BALP detection kits. All steps had to be conducted according to instructions.

### 2.6. Western Blot

The samples of mouse joint synovium were collected, and RIPA lysis buffer was applied to collect the total protein. After protein quantification, 20 *μ*g protein was taken to conduct 10% SDS-PAGE, and then was transferred to PVDF membranes. With blocking solution sealed at ambient temperature for 2 h, the membranes were incubated with rabbit monoclonal antibodies p-IKK*β* (1 : 1000, ab38515), p-I*κ*B*α* (1 : 1000, ab13362), p50 (1 : 1000, ab32360), and rabbit polyclonal antibody GAPDH (1 : 1000, ab9485) overnight at 4°C. On the second day, the membranes were washed by PBST and then incubated with HRP-labeled secondary antibodies at room temperature for 1 h. Subsequently, PBST was utilized to wash membranes for 1 h. Finally, enhanced ECL Chemiluminescence Detection Kit was applied to check target protein. The gray value was analyzed by ImageJ software.

### 2.7. Statistical Analysis

Each experiment was repeated three times. Measurement data was expressed by mean ± standard deviation (SD). Statistical analysis was evaluated by SPSS 22.0 software (SPSS, Inc., Chicago, IL, USA). The comparison between the two groups was tested by Student's *t*-test. A statistically significant difference was suggested if *P* < 0.05.

## 3. Results

### 3.1. Effects of PD-1 and OX40 on CIA Mouse Arthritis Score and Pathology of Joint Tissues

The result of arthritis score indicated that, compared with the control group, mice arthritis scores in the CIA group were higher; compared with the CIA group, mouse arthritis scores in the PD-1-Fc group were upregulated while arthritis scores in the OX40-Fc group was downregulated. Mice arthritis scores in the PD-1-Fc + OX40-Fc group were higher than that in the OX40-Fc group (Figure 1(a), *P* < 0.05).

HE staining results suggested that the cartilage tissues of mice were normal in the control group. In the CIA group, cartilage tissues structure were damaged, and chondrocytes were arranged loosely; pyknosis and apoptosis occurred in a small amount of chondrocyte nucleus; a large number of inflammatory cells were infiltrated, neovascularization was conducted, and the articular surface seriously damaged. The pathological score of the CIA group was significantly higher than that in the control group. Compared with the CIA group, pathological changes were aggravated in the PD-1-Fc group; the latter group showed that cartilage tissues structure was damaged seriously, chondrocytes were in apoptosis, synovial cells proliferated, and the surface of joints got rough and pathological score increased rapidly. Compared with the CIA group, in the OX40-Fc group, a significant decrease was occurred in the destruction of cartilage structure of ankle joint, inflammatory cell infiltration, synovial hyperplasia, and neovascularization as well as pathological score. Compared with the OX40-Fc group, in the PD-1-Fc + OX40-Fc group, the destruction of cartilage tissues was aggravated, synovial hyperplasia and neovascularization increased, and the pathological score increased quickly (Figures 1(b) and 1(c)).

The article "OX40-Fc Fusion Protein Alleviates PD-1-Fc-Aggravated Rheumatoid Arthritis by Inhibiting Inflammatory Response" was retracted in 2023. Reasons: signs of a paper mill; suspected computer-generated content; unreliable results or conclusions; concerns about the data.

Above results indicated that PD-1-Fc could promote arthritis damage in CIA mice, while OX40-Fc could reverse this effect.

### 3.2. Effects of PD-1 and OX40 on Immune Molecules in PBMC Peripheral Blood of CIA Mouse

The result of flow cytometry suggested that, compared with the control group, the proportion of CD4+ T cells and CD28+ positive cells in PBMCs of CIA group mice decreased significantly, while the proportion of CD8+ T cells and CD19+ cells increased rapidly. PD-1-Fc could promote the reduction and increase of immune molecules in PBMCs of CIA mouse; but OX40-Fc could increase the proportion of CD4+ T cells and CD28 + positive cells and reduce the proportion of CD8+ T cells and CD19+ cells in CIA mouse. Besides, compared with the PD-1-Fc group, proportion of PD-1-Fc-caused immune molecules in PBMC was reversed in the PD-1-Fc + OX40-Fc group (Figures 2(a) and 2(b), *P* < 0.05).

### 3.3. Effects of PD-1 and OX40 on Inflammatory Factor Levels in Serum of CIA Mouse

The effects of PD-1 and OX40 on inflammatory factors in CIA mouse were further detected by ELISA. The result indicated that, compared with the control group, the level of CRP, IL-2, IL-4, IL-1*β*, and INF-*γ* in the serum of CIA group increased significantly. Compared with the CIA group, the level of CRP, IL-2, IL-4, IL-1*β*, and INF-*γ* in PD-1-Fc rose up quickly in the PD-1-Fc group while in the OX40-Fc group, it downregulated rapidly. However, PD-1-Fc combined with OX40-Fc could significantly downregulate the level of inflammatory factors in the PD-1-Fc group (Figures 3(a)–3(e), *P* < 0.05). The result suggested that OX40-Fc could inhibit PD-1-Fc-aggravated inflammatory response of CIA mouse.

### 3.4. Effects of OX40-Fc and PD-1-Fc on Markers of Bone Metabolism in CIA Mouse

Markers of bone metabolism (CTX-I and TRACP-5b) in mice were measured by ELISA (Figures 4(a)–4(c)). The result confirmed that, compared with the control group, the levels of CTX-I and TRACP-5b in synovium of the CIA group increased significantly, and the level of BALP decreased rapidly (*P* < 0.05). PD-1-Fc could significantly promote the levels of CTX-I and TRACP-5b, but reduce the level of BALP in CIA mice (*P* < 0.01). However, OX40-Fc significantly inhibited CTX-I and TRACP-5b levels and upregulated BALP levels in CIA mice (*P* < 0.05). Additionally, compared with the OX40-Fc group, the levels of CTX-I and TRACP-5b in the PD-1-Fc + OX40-Fc group increased significantly, while the level of BALP decreased significantly (*P* < 0.05). The result suggested that OX40-Fc could inhibit PD-1-Fc-aggravated bone metabolism in synovium tissues of CIA mice.

The article "OX40-Fc Fusion Protein Alleviates PD-1-Fc-Aggravated Rheumatoid Arthritis by Inhibiting Inflammatory Response" was retracted in 2023. Reasons: signs of a paper mill; suspected computer-generated content; unreliable results or conclusions; concerns about the data.

### 3.5. Effects of OX40-Fc and PD-1-Fc on NF-*κ*B Signal Pathway in Synovium Tissues of CIA Mice

Studies suggested that NF-*κ*B signal pathway was regarded as one of the main inflammatory pathways in RA [27]. Therefore, NF-*κ*B pathway proteins (p-IKK*β*, p-I*κ*B*α* and p50) were detected by western blot to determine relevant molecular mechanism. The result indicated that (Figures 5(a) and 5(b)), compared with the control group, the protein expression of p-IKK*β*, p-I*κ*B*α*, and p50 in synovial tissues of the CIA group was significantly increased (*P* < 0.01). Compared with the CIA group, the protein expression of p-IKK*β*, p-I*κ*B*α*, and p50 in the PD-1-Fc group increased significantly while in the OX40-Fc group, all expression was a significant decrease (*P* < 0.01). Besides, the protein expression in the PD-1-Fc + OX40-Fc group was significantly lower than that in the PD-1-Fc group, while higher than that in the OX40-Fc group (*P* < 0.01). The result indicated that the OX40-Fc inhibited the activation of PD-1-Fc-aggravated NF-*κ*B pathway in synovial tissues of CIA mice.

## 4. Discussion

RA is a T cell-mediated autoimmune disease, and PD-1 as well as OX40 costimulation signals plays an important role in regulating the activation of CD4 + T cells. Abnormal costimulation signals are associated with a variety of autoimmune diseases [28]. Abnormal PD-1 and OX40 signals lead to the changes of T cell biological behavior [29, 30]. In researches on animal models, loss or blocking of PD-1 signal can cause a series of autoimmune diseases [31, 32], while knockout or blocking of OX40 signal can treat autoimmune diseases to some extent [33]. CD4 + PD-1+ and CD4 + OX40+ T lymphocytes were enriched in the synovial fluid of RA patients [34], suggesting that abnormal PD-1 and OX40 signals are involved in the immunopathological process of RA. However, in RA patients, the expression of PD-1 and loss of CD28 do not clear autoreactive T cells to maintain the balance of costimulation signals in autoimmunity [35]. It is concluded that an imbalance between negative PD-1 and positive OX40 costimulation signals may be existed in RA immunopathology. This imbalance promotes the abnormal activation of CD4+ autoreactive T cells, induces autoimmunity, and then causes diseases to be delayed healing [24]. In this paper, OX40-Fc and PD-1-Fc fusion proteins were used to intervene the CIA mouse model. The results indicated that OX40-Fc could improve arthritis while PD-1-Fc-aggravated arthritis in CIA mice; OX40-Fc could reduce the destruction of articular cartilage tissue structure and inflammatory cell infiltration, while PD-1-Fc could destroy the repair effect of OX40-Fc on RA mice. The results suggested that abnormal costimulation signals of PD-1 and OX40 may play an important role in the pathological process of AR.

The article "OX40-Fc Fusion Protein Alleviates PD-1-Fc-Aggravated Rheumatoid Arthritis by Inhibiting Inflammatory Response" was retracted in 2023. Reasons: signs of a paper mill; suspected computer-generated content; unreliable results or conclusions; concerns about the data.

In this study, CD4 + T cells played a critical role in mediating the onset of arthritis, the occurrence of autoantibodies, and the progression of synovitis. It was found that when the proportion of CD4+ T cells in PBMCs of CIA mice decreased, the proportion of CD8+ T cells increased. The reason may be that in the process of chronic inflammation of RA joint, a large number of CD4+ T cells migrate and infiltrate into inflammatory sites in peripheral blood, resulting in the decrease of depletion of this T cell subset in peripheral blood of patients, while the decrease of CD4+ T cells leads to a relatively higher proportion of CD8+ T cells [36, 37]. As a representative costimulation molecule of the B7 family, the CD28 expression is mainly on the surface of T cells and bonds with B7 on the surface of APCs to initiate the activation of T cells. In order to study the changes of the costimulatory molecule expression in RA patients, the expression of CD28 was detected first; it was found that the expression of CD28 decreased significantly in CIA mouse model, suggesting that some T cells might lose the expression of CD28 during the immune process of RA. After the intervention to OX40-Fc and PD-1-Fc fusion protein, the proportion of CD4 + T and CD28+ cells increased significantly while in CD8 + T and CD19+ cells, there was a significant decrease in the OX40-Fc group. Compared with the PD-1-Fc group, the proportion of CD4 + T and CD28+ cells in the PD-1-Fc + OX40-Fc group was increased significantly, while in CD8 + T and CD19+ cells, there was a significant reduction. The results indicated that OX40-Fc could intervene PD-1-Fc-induced destruction of immune system in CIA mice.

The article "OX40-Fc Fusion Protein Alleviates PD-1-Fc-Aggravated Rheumatoid Arthritis by Inhibiting Inflammatory Response" was retracted in 2023. Reasons: signs of a paper mill; suspected computer-generated content; unreliable results or conclusions; concerns about the data.

In addition, CD4+ Th cells are adaptive immune cells that release proinflammatory cytokines (IFN-*γ*, IL-6, IL-17) or anti-inflammatory cytokines (IL-4, IL-10, IL-13) to regulate cellular and humoral immune responses [38, 39]. Abnormal differentiation is the main cause of RA immune imbalance, and the plasticity of differentiation may cause repeated disturbance of RA immune balance, especially when abnormal differentiation produces a large number of inflammatory factors (CRP, IL-2, IL-4, IL-1*β*, INF-*γ*) [40, 41]. In this study, these inflammatory factors were detected by ELISA in different groups of mice, and the result revealed that the serum levels of CRP, IL-2, IL-4, IL-1*β*, and INF-*γ* were significantly increased in the CIA group and further increased in the PD-1-Fc group, while OX40-Fc significantly reduced the levels of these factors; meanwhile, OX40-Fc could reverse the PD-1-Fc-aggravated inflammation in CIA mice.

Abnormal bone metabolism and activation of NF-*κ*B signaling pathway are also manifestations of RA [27, 42]. Liang et al. found that silencing ZNRF3 attenuated knee injury and reduced inflammation levels in CIA mice, which was associated with inactivation of the NF-*κ*B signaling pathway [43]. In this study, the contents of bone metabolism-related genes CTX-I and TRACP-5b and the expression of NF-*κ*B signaling pathway-related proteins (p-IKK*β*, p-I*κ*B*α*, p50) in synovium of the CIA group were further determined. PD-1-Fc fusion protein aggravates abnormal bone metabolism and inflammatory response in RA, while OX40-Fc fusion protein can significantly inhibit the occurrence of the above pathological conditions, and has a reversal effect on the exacerbation caused by PD-1. However, it has been found that activated NF-*κ*B has a dual role in promoting or inhibiting inflammation, which is closely related to its upstream stimulators and downstream activators [44]. This needs to be confirmed by our further experimental studies. Additionally, since the synovial tissue and serum samples in the CIA mice model were detected in this study, they could not fully represent the real situation of clinical patients, and PD-1 and OX40 molecules on the cell surface were not detected. Therefore, this experiment needs to be further studied.

In conclusion, OX40-Fc was confirmed to significantly reverse arthritis injury in CIA mice exacerbated by PD-1-Fc. This verification provides biological markers with clinical significance for the diagnosis and prognosis of RA. At the same time, it also offers theoretical and experimental basis to new immune intervention targets.

## Figures and Tables

**Figure 1:** Effects of PD-1 and OX40 on CIA mice arthritis score and pathology of joint tissues. (a) The arthritis scores of each group. (b) Histopathological changes of mice ankle joints in groups. (c) Histopathological score of mice ankle joints in each group. ^∗^*P* < 0.05 and ^∗∗^*P* < 0.01. CIA: collagen-induced arthritis.

The article "OX40-Fc Fusion Protein Alleviates PD-1-Fc-Aggravated Rheumatoid Arthritis by Inhibiting Inflammatory Response" was retracted in 2023. Reasons: signs of a paper mill; suspected computer-generated content; unreliable results or conclusions; concerns about the data.

**Figure 2:** Effects of PD-1 and OX40 on immune molecules in PBMC peripheral blood of CIA mice. (a) Flow cytometry was utilized to detect proportion of CD4 + T, CD8+ T, CD28+, and CD19+ cells in PBMC peripheral blood in groups. (b) Proportion of CD4+ T, CD8 + T, CD28+, and CD19+ positive cells was qualified and analyzed. ^∗^*P* < 0.05 and ^∗∗^*P* < 0.01. PBMC: peripheral blood mononuclear cell.

**Figure 3:** Effects of PD-1 and OX40 on inflammatory factor levels in serum of CIA mice. The level of CRP (a), IL-2 (b), IL-4 (c), IL-1*β* (d), and INF-*γ* (e) in serum was measured by enzyme linked immunosorbent assay (ELISA). ^∗^*P* < 0.05 and ^∗∗^*P* < 0.01.

**Figure 4:** Effects of OX40-Fc and PD-1-Fc on markers of bone metabolism in CIA mice. The levels of CTX-I (a), TRACP-5b (b), and BALP (c) in synovial tissues of mice in each group were detected by ELISA. ^∗^*P* < 0.05 and ^∗∗^*P* < 0.01.

**Figure 5:** Effects of OX40-Fc and PD-1-Fc on NF-*κ*B signal pathway in synovium tissues of CIA mice. The protein expression of p-IKK*β*, p-I*κ*B*α*, and p50 in synovial tissues of mice in each group was detected by Western blot. ^∗^*P* < 0.05 and ^∗∗^*P* < 0.01.

## Data Availability

The data used to support the findings of this study are available from the corresponding author upon request.
